# Sports Training System Based on Convolutional Neural Networks and Data Mining

**DOI:** 10.1155/2021/1331759

**Published:** 2021-09-20

**Authors:** Yuwang Zhang, Yuan Zhang

**Affiliations:** Department of Physical Education, China University of Geosciences (Beijing), Beijing 100083, China

## Abstract

In recent years, China's sports industry has achieved good development, but the efficiency of athletes in the training process is difficult to have scientific guarantee. How to use scientific algorithm and data mining technology to accurately guide the sports training process has become a hot spot. Based on this, this paper studies the gait recognition model of sports training based on convolutional neural network algorithm. First, this paper analyzes the research status of gait recognition in the process of training and optimizes and improves the deficiencies in sports training. Then, the convolutional neural network algorithm and data mining technology are optimized and analyzed in the gait recognition model. Finally, the experimental results show that the convolutional neural network algorithm can realize the recognition and model reconstruction of athletes' gait in the training process and can make the optimal strategy according to the gait differences of different athletes in the training process, and the recognition accuracy of athletes' gait can reach more than 97%.

## 1. Introduction

At present, there are some problems in the daily training process, such as single training method long-term training leading to bone and joint injury. [1]. How to recognize the gait of athletes through the existing intelligent algorithms and then help athletes correct their posture in the training process has become a hot spot [2]. In addition, when athletes perform these actions in training or competition, each joint of the human body has different angles, and the change of these angles will affect the effect of action, thus affecting the play of these skills [3]. Because of the competitive nature of most sports, people in the process of sports cannot avoid collision and can easily experience sports injury [4]. In the daily sports training process, there are few professional auxiliary systems or tools for high-precision collection and intelligent analysis of human body data during exercise [5]. Therefore, if the athlete's gait and limb movements are simulated and predicted, this can play an important role in the training of sports skills and the prevention of sports injuries [6].

At present, there are many research directions on gait recognition of sports athletes. Some scholars have studied training methods, gait recognition models, gait prediction, and the combination of gait recognition and artificial intelligence [7]. Landgraff et al. combined the convolutional neural network model to intelligently optimize the current sports training system, highlighting the acquisition of data from sensors, and realizing intelligent control of the sports training system according to specific indicators [8]. In order to improve the training efficiency of athletes in the daily training process and make full use of the data information in the training process, Hassib et al. chose a convolutional neural network algorithm to analyze the data of two groups of different teams in the competition. This study confirmed the effectiveness of this method in guiding athletes during basketball games [9]. According to the idea of convolutional neural network, Tafti et al. studied the track diameter, transportation weight, safety performance, and resistance of the sphere in sports and intelligently obtained various parameters and influencing factors in the process of sports training system [10]. Ramesh et al. combined the factors affecting sports training with the athlete's gait recognition process, combined with neural network algorithms, to study the influence of gait recognition on sports performance [11]. Luan studied the coupling relationship between the sphere's motion trajectory and the athlete's gait and finally combined with the convolutional neural network algorithm and designed experiments to prove the role of this method in improving the safety of basketball [12]. Talasila et al. have studied the factors that have a greater impact on the sports training process by combining multiple neural network analysis strategies and selected superresolution factors to establish a functional relationship between gait recognition and different dynamic performance [13]. Hu et al. have found that sports have a problem of low resolution during training. They have completed the multidimensional application of different data and information by setting up a variety of control experiments [14]. Xie and Grossman have confirmed the effectiveness and feasibility of convolutional neural networks in the process of sports judgment, and the research results can also provide a basis for the safety of basketball in various environments [15]. Prusa and Khoshgoftaar conducted modeling and analysis on the training process data of different types of sports, compared the data analysis conditions required for different types of sports through convolutional neural network models, and evaluated them by observing different experimental data [16]. Lee et al. integrated data on the multiple gaits of athletes in different sports, used convolutional neural network models to analyze the forces, and evaluated the safety of athletes' multiple gaits in different sports with reference to relevant standards [17]. Chen and Jahanshahi analyzed the application of different algorithms in sports and found that, in the training data analysis link of football sports, the difference dialectical method based on the convolutional neural network algorithm was used for data analysis and found that this method has more advantages [18]. Kim et al. have conducted various studies on the recognition effect of key training nodes in the process of basketball players adopting different styles of training programs and introduced the particle swarm optimization algorithm for optimization evaluation [19]. Sun et al. proposed a convolutional neural network algorithm based on Bernoulli matrix. The results show that the algorithm can reduce the problem of gait recognition of sports athletes during dynamic movement, but it reduces the accuracy of partial recognition [20]. In order to improve the recognition accuracy, Nguyen et al. proposed an optimization model for dislocation gait recognition based on ant colony algorithm and particle swarm algorithm. The effectiveness of the model was verified by design experiments [21]. Xiao et al. created a dynamic motion map by simulating the gait of sports athletes, achieving accurate recognition of athletes' gait, and improving the intelligence of sports athletes' gait recognition [22].

In summary, it can be found that, among the existing research results, its innovations mainly focus on the application of intelligent algorithms, such as convolutional neural network algorithms or particle swarm algorithms to sports training systems, but they are only simple applications and cannot be mined from data. From the perspective of in-depth analysis and utilization of the data generated by the sports training system, the constructed sports' training system has problems, such as poor reliability, small application range, weak intelligence, and low data utilization [23]. On the other hand, research has not focused on the research and model construction of sports training systems based on convolutional neural network algorithms and data mining techniques [24]. Aiming at the problem of “only simple migration and application of intelligent algorithms, but not deep mining of the value of data” existing in the latest research, research on sports training systems based on convolutional neural networks and data mining has important practical significance.

The contribution made by this paper is as follows. An improved convolutional neural network algorithm is proposed, which can realize not only the intelligent acquisition and classification of the data generated by the sports training system, but also the effective information contained in the data. On the basis of roughly recognizing the gait of athletes during training, it can make full use of data mining technology to realize the dynamic modeling of real athletes' gait by making full use of the spatial video and image sensing information and use the extremes of multivariate functions. The numerical value is used to quantitatively describe the similarity and consistency between each comparison column (training effect on target athletes) and reference column (known effective information of athlete's gait during training), so as to quantify the training effect of target athletes. The weight ranking can make full use of the gait recognition information of each sports athlete to achieve accurate modeling and simulation of the training process.

In order to solve the problem of intelligent acquisition and efficient use of data in the sports training system, this paper studies the sports training system, which is mainly divided into four parts.  Section 1 introduces the current status of gait recognition technology and training system in sports athletes.  Section 2 introduces the application idea of convolutional neural network in sports training system.  Section 3 builds an athlete's gait recognition model based on the convolutional neural network algorithm and proposes an optimization model for sports training gait recognition based on Gaussian random distribution and constructs a sports training system based on data mining and gait recognition.  Section 4 discusses the experimental results and analyses on the sports training gait recognition model constructed in this paper.  Section 5 draws conclusions.

## 2. Application of Convolutional Neural Network in the Sports Training System

The learning paradigm of convolutional neural networks (CNN) can be divided into supervised learning and unsupervised learning [25, 26]. In this study, through the deep learning of individual characteristics, gait tracking, and training environment among athletes, the construction of training gait recognition model based on convolutional neural network algorithm is realized. First, the convolutional neural network algorithm is selected, and three parameters related to the gait recognition of athletes are selected to design an athlete gait recognition system based on convolutional neural network algorithm. Then, through the research on the monitoring process of athletes' gait, morphological time, and three-dimensional reconstruction conditions, the hierarchical framework and index relationship of the whole intelligent gait recognition system are designed, and the control of the key conditions of the gait recognition system is refined from multiple angles. Second, convolutional neural network algorithm and data mining technology are used to test its accuracy.

In this paper, the multilayer convolutional neural network algorithm structure is used in the sports training system for a certain sports event and the training information intelligent processing model based on existing athletes. It is assumed that the first input value of the target, the implicit input value of the security feature, the output layer data of the security judgment, and the number of its nodes are known. In addition, in the force simulation of the Hybrid III crash dummy model, the crash dummy model has the characteristics of force, and its algorithm includes joint friction, nonlinear stiffness, damping, and joint range of motion in the process of gait. The joint moment is based on the stiffness, damping, and friction coefficient data measured by Armstrong Aerospace Medical Laboratory. According to the international adult body size standard, the live load is calculated as 750 N/person, the weight of the mannequin is 75 kg, the height is 175 cm, and the age is 20. The specific parameters of the manikin are shown in Table 1.

## 3. Sports Training System Based on Convolutional Neural Network and Data Mining

### 3.1. Gait Recognition Model of Sports Athletes Based on Convolutional Neural Networks and Data Mining

In the current mainstream research, gait recognition models based on motion process and cosimulation process are mainly divided into basic model and structural model, in which the basic model includes sequential model and parallel model, and the structural model includes cyclic model. This study uses convolutional neural network algorithm (CNN) to simulate and analyze the athlete's gait modeling process. In this process, the convolutional neural network algorithm first performs data-level binarization of different data types, filters them, and eliminates gross errors in combination with the judgment function; second, it combines the characteristics of different types of athletes. Multiple representations of different types of arrays are realized, and their data fit is further differentiated. In addition, in the analysis process of different sports training arrays, the number of convolutions and the number of neural network layers are different, and they will be different from different types. The data group is related, so information mining is needed. The key of data mining is to distinguish between different data groups according to the threshold judgment standard. After distinguishing, in order to identify and judge the training data for the first time, the analysis of different types of data groups is realized. According to the characteristics of convolutional neural network and data mining, its principle is shown in Figure 1.

The conventional CNN model can extract the key data of sports training through multiple convolution training processes, but it is easy to ignore the distinction between different types of data groups, and it is easy to make wrong judgments on data that appears multiple times in the same data group, making the key information of the data group inaccurate. If we continue to use the conventional CNN model to express the coupling relationship between human resources and other resources, it will cause the lack of process information and make the simulation results inaccurate. In view of this situation, it is necessary to extend the conventional CNN model, that is, to model by multivalued CNN model. The multidimensional matrix is used to describe the calculation cycle, order coupling degree, and resource coupling degree in the design process, which is called multivalued CNN model. The coupling degree function *Q*(*x*) and the period function *T*(*x*) are as follows:

(1) $$\begin{array}{c} Q\left(x\right)=\frac{x^{4}+7x^{3}+\sqrt{\left|5x^{2}+2x\right|}}{5x^{3}+3x^{2}+\sqrt{\left|x+x^{-1}\right|}},\\ T\left(x\right)=\frac{8x^{4}+6x^{3}+3x^{2}+2}{\sqrt{7t^{3}+9t^{2}+1}}, \end{array}$$

where *x* is the original data input in each movement process and *t* is the single cycle training calculation cycle.

In the application process of this research, the CNN model needs to be self-learning through some datasets. In the learning process, because the time difference of different cosimulation processes is very large. It is determined in advance that the information includes the number of convolutions and data dimension information. In the CNN model, the learning process of the convolution processing of the data is shown in Figure 2.

According to the definition of neuron node, the single value of the period of different dimensions is *t*, and the total number of analysis times is *n*. Through the single value of different periods and the period judgment of the entire data analysis process, the calculation period of different types of data can be determined. At this time, the calculation period is as follows:

(2) $$\begin{array}{c} T{}^{\prime }\left(x\right)=\frac{8x^{4}+6x^{3}+3x^{2}+2}{\sqrt{4n^{3}+3n^{2}+7n+3}+\sqrt{7t^{3}+9t^{2}+1}}. \end{array}$$

According to the sequence dependence relationship between two process nodes, the judgment function is as follows:

(3) $$\begin{array}{c} P\left(x\right)=1-\left|\frac{\sqrt{7x^{4}+8x^{3}+3x^{2}+9}}{\sqrt{4n^{4}+3n^{3}+7n+3}+\sqrt{9x^{3}+3x^{2}+1}}\right|. \end{array}$$

After the first convolutional neural network analysis, the single output function is as follows:

(4) $$\begin{array}{c} H\left(x\right)=\frac{3x^{4}+2x^{3}+5x^{2}+1}{3x^{3}+3x^{2}+1}, \end{array}$$

where *x* represents the original data of each motion process and *n* represents the single cycle motion process node.

### 3.2. Simulation Modeling of Gait and Ankle Joint Changes of Jump Shot Touchdown in Sports Training

First, this paper simulates the touch action of jump shot in the process of training. It simulates the physical condition of the athlete and the gait data information. The process of simulation analysis is shown in Figure 3.

At the moment of landing, the gait of different athletes presents different physical changes, which is not strong. Because of the individual differences between each athlete, there are also differences in the experimental process and the simulation modeling process between different athletes. Therefore, in the process of analyzing the intensity of the sports training process for different types of datasets, the coupling functions and standardized values used are also different. This study first collected a large number of sports data performed by athletes in different environments and at different time periods (such as morning exercises, evening exercises, and professional exercises) as training samples, combined with convolutional neural network algorithm. The deep-level information included in the data is analyzed many times to realize the three-dimensional reconstruction of different athletes' postures, so as to help the athletes' steps. This improves the effect and accuracy of state recognition. The reference values are shown in Table 2.

On the other hand, in order to further reduce data mining errors, we also established a basic gait recognition database in the process of experiment to realize continuous updating and correction. The data updating process is shown in Figure 4.

The CNN sports training gait recognition optimization analysis model designed in this research adopts the processing method to combine the safe gait feature comparison data generated by the gait of different athletes and synthesize a new set of behavior feature vectors. In the process of analyzing the data, it will perform the first round of prejudgment based on the characteristics of different types of data groups and the set threshold differences of different types. According to the judgment results, the corresponding feature vectors are marked. The value of multidimensional sports training information is compared to determine the best factor matching rate. After these values are determined, the stability of different types of data can also achieve multilevel discrimination and analysis of these processes, so overall, the process has a higher utilization rate and stability. The processing process of sports training data based on convolutional neural network and data mining technology is shown in Figure 5.

## 4. Result Analysis and Discussion

### 4.1. Verification Experiment of the Sports Training System Based on Convolutional Neural Network Algorithm and Data Mining

Considering that the gait of athletes in different sports is different, it is necessary to add different training conditions for athletes in different sports before the formal experiment, so as to avoid the data misjudgment in the process of athletes' training. The parameter settings in the experiment process are shown in Table 3.

In the process of the experiment, the gait recognition constraints of different athletes will be realized through the following three aspects. First, the common training gait of known sports is decomposed and expressed and stored in the form of matrix. In this way, the dynamic changes and recognition of the gait of different athletes can be realized. In the link of analyzing and coupling the data, first, through the convolutional neural network algorithm, the multidimensional information is extracted from the initial data generated during the experiment. Then compare the mining and analysis results of different types of experimental data with standard sports training reference values. After analyzing these data results, compare the different types of data results and classify them according to the training rules.

Second, by solving the feature vectors of different gait vectors and multiplying the dot products, the athletes will be tested in multiple dimensions, including video detection, image detection, and motion trajectory tracking detection. In the detection process, by setting different constraint thresholds according to different sports items, the data to be tested are input into the convolutional neural network training system, and the analyzed data results obtained are compared with features, and then, compare it with the standard reference value. After completing these links, analyze the similarity of the data generated by these sports training systems and perform clustering processing.

Finally, after analyzing different types of experimental data, perform multiple error analyses until the minimum requirements set are met. The final results can be output. The experimental data and preliminary experimental results are shown in Figure 6.

It can be seen from Figure 6 that the exercise training system using convolutional neural network and data mining method is more reliable than the exercise training system using genetic programming neural network (GP-NN) and simple data mining method, and its maximum value is 93, and its data change law is more in line with the change trend of Bernoulli function.

### 4.2. Experimental Results and Feedback Analysis

This paper conducts a confirmatory experiment on multiple sets of training data and, according to the differences of the experimental data, conducts multiple experiments on different types of sports data (basketball, football, etc.). In order to make the experimental results more accurate, random factors are used to simulate the reality. The different factors in the situation and the error of the function are repaired and verified through a large number of public data samples. The error analysis results are shown in Table 4.

Finally, compared with the latest research methods (neural network model represented by CNN algorithm and data mining model represented by nonlinear analysis), the experimental results show that the convolutional neural network algorithm model can realize the verification and error analysis of the function in the gait prediction of athletes in training and also verify the effectiveness and feasibility of the model, so the model can also provide the basis for the gait analysis of sports training in various environments. In addition, among the results obtained by using convolutional neural networks and data mining methods, the comparative analysis of take-off height (i.e., weight deviation fluctuation) without fatigue shows that fatigue has a significant impact on take-off height, and the training degree of the subjects who are already tired is much lower than the reference value (*p* < 0.001). This shows that, in this process, compared with the latest research methods (the neural network model represented by the CNN algorithm and the data mining model represented by the nonlinear analysis), the CNN-DM model is not only better than the current mainstream research results. The accuracy is high, and it can accurately recognize the athlete's gait during the training process. It can detect the rotation angle of the ankle joint and the training effect. The experimental analysis results are shown in Figure 7.

It can be seen from Figure 7 that, among the results obtained by the three different training methods, the error rate of training and gait recognition in the group using convolutional neural network algorithm is significantly lower than that using conventional neural network algorithm. Convolutional neural network and data mining have been used in the training system. With the increase of training times, the accuracy of experimental results shows a convergence trend. When the number of training times reaches a certain number, the change of error degree is very small, and the data accuracy can reach 97.5%.

## 5. Conclusion

In recent years, China's sports industry has developed well, but the efficiency and data utilization in the process of sports training need to be further improved. How to use a scientific algorithm for accurate guidance has become a hot spot. Based on this, in order to solve the problem of intelligent acquisition and high-efficiency use of data in the sports training system, this paper studies the sports training system. Compared with the latest research results at this stage, the method proposed in this research can achieve the effect of sports training. The data generated by the training system can be obtained and classified intelligently, and the effective information contained in the data can be deeply mined, and the error rate is lower. First, this paper analyzes the research status of gait recognition, optimizes and improves the shortcomings of the current research hotspot in gait recognition, and then optimizes and analyzes the convolutional neural network algorithm in gait recognition model. Finally, the experimental results show that the sports training system based on convolutional neural network algorithm can realize the recognition and model reconstruction of athletes' gait in the training process and can make the optimal strategy according to the differences of different athletes' gait in the training process, and the gait recognition accuracy can reach more than 97%. However, this paper only focuses on the gait recognition of sports athletes in the process of competition and does not take the potential impact of different gait of sports athletes into consideration. Therefore, the comprehensive analysis and evaluation of this index system need to be further studied.

## Figures and Tables

**Figure 1:** Data processing principle based on convolutional neural network algorithm.

**Figure 2:** The convolution processing process of the CNN model on the data.

**Figure 3:** The process of simulating and analyzing athlete characteristic data.

**Figure 4:** Data update process of gait recognition database.

**Figure 5:** Data processing based on convolutional neural network and data mining.

**Figure 6:** Model flow under constraints.

**Figure 7:** Experimental result output curve.

**Table 1:** Human body morphologic parameters.

Parameter name	Parameter
Age (months)	240
Weight	75 kg
Standing height	175 cm
Left shoulder Ht.	56.309
Right	18.987
Left	18.968
Live load	750 N

**Table 2:** Gait recognition effect and accuracy reference value.

Reference indicator	Reference
Gait posture	0.22 ± 0.01
Gait movement	0.21 ± 0.01
Gait stability	0.34 ± 0.01
Gait training standard	0.16 ± 0.01
Gait sensing accuracy	0.18 ± 0.01

**Table 3:** Parameter settings during the experiment.

Experimental parameters	Reference
Neural network layer	5
Data mining times	10
Data coupling center	4
Error control	0.5
Number of gait training models	20

**Table 4:** Experimental error analysis results.

Error index	Before optimization	Optimized	Degree of error
Data mining and convolutional neural network group	0.21 ± 0.005	0.15 ± 0.005	<0.001
Neural network experimental group	0.26 ± 0.005	0.19 ± 0.005	<0.002
Single-level convolutional neural network algorithm group	0.25 ± 0.005	0.18 ± 0.005	<0.001

## Data Availability

The data used to support the findings of this study are available from the corresponding author upon request.

## References

[1] Babio G. D., Janavel G. V., Constantin I. (2021). Atrial size and sports. a great training for a greater left atrium: how much is too much. *The International Journal of Cardiovascular Imaging*.

[2] Wang T., Chen Y., Qiao M., Snoussi H. (2018). A fast and robust convolutional neural network-based defect detection model in product quality control. *International Journal of Advanced Manufacturing Technology*.

[3] Halén P., Khan K. M. (2019). Finland’s sports physiotherapy conference-athlete training and loading: Helsinki 7-8 June 2019. *British Journal of Sports Medicine*.

[4] Emery C. A., Berg C., Richmond S. A. (2019). Implementing a junior high school-based programme to reduce sports injuries through neuromuscular training (iSPRINT): a cluster randomised controlled trial (RCT). *British Journal of Sports Medicine*.

[5] Morgenlander J. C., Hainline B. (2018). Emerging Subspecialties in neurology: sports neurology training and certification: an overview in 2018. *Neurology*.

[6] Chu W. C.-C., Shih C., Chou W.-Y., Ahamed S. I., Hsiung P.-A. (2019). Artificial intelligence of things in sports science: weight training as an example. *Computer*.

[7] Hu H., Tang B., Gong X., Wei W., Wang H. (2017). Intelligent fault diagnosis of the high-speed train with big data based on deep neural networks. *IEEE Transactions on Industrial Informatics*.

[8] Landgraff H. W., Riiser A., Lihagen M., Skei M., Leirstein S., Hallén J. (2021). Longitudinal changes in maximal oxygen uptake in adolescent girls and boys with different training backgrounds. *Scandinavian Journal of Medicine & Science in Sports*.

[9] Hassib E. M., El-Desouky A. I., Labib L. M., El-kenawy E.-S. M. (2020). WOA + BRNN: an imbalanced big data classification framework using whale optimization and deep neural network. *Soft Computing*.

[10] Tafti A. P., Badger J., LaRose E. (2017). Adverse drug event discovery using biomedical literature: a big data neural network adventure. *JMIR Medical Informatics*.

[11] Ramesh V. P., Baskaran P., Krishnamoorthy A., Damodaran D., Sadasivam P. (2019). Back propagation neural network based big data analytics for a stock market challenge. *Communications in Statistics—Theory and Methods*.

[12] Luan Z. (2019). The effect of beach sports power training on ankle joint injury. *Journal of Coastal Research*.

[13] Talasila V., Madhubabu K., Madhubabu K., Mahadasyam M., Atchala N., Kande L. (2020). The prediction of diseases using rough set theory with recurrent neural network in big data analytics. *International Journal of Intelligent Engineering and Systems*.

[14] Hu H., Liu Z., An J. (2020). Mining mobile intelligence for wireless systems: a deep neural network approach. *IEEE Computational Intelligence Magazine*.

[15] Xie T., Grossman J. C. (2018). Crystal graph convolutional neural networks for an accurate and interpretable prediction of material properties. *Physical Review Letters*.

[16] Prusa J. D., Khoshgoftaar T. M. (2017). Improving deep neural network design with new text data representations. *Journal of Big Data*.

[17] Lee K. Y., Kim K. H., Kang J. J. (2017). Comparison and analysis of linear regression & artificial neural network. *International Journal of Applied Engineering Research*.

[18] Chen F. C., Jahanshahi R. (2018). NB-CNN: deep learning-based crack detection using convolutional neural network and naïve bayes data fusion. *IEEE Transactions on Industrial Electronics*.

[19] Kim K. S., Lee S., Huang K. (2018). A scalable deep neural network architecture for multi-building and multi-floor indoor localization based on Wi-Fi fingerprinting. *Big Data Analytics*.

[20] Sun Y., Szűcs G., Brandt A. R. (2018). Solar PV output prediction from video streams using convolutional neural networks. *Energy & Environmental Science*.

[21] Nguyen T., Bui V., Nehmetallah G. (2018). Computational optical tomography using 3-D deep convolutional neural networks. *Optical Engineering*.

[22] Xiao L., Liu W. Y., Lin P. Z., Guo G.-C., Zhang Y.-S., He L. (2018). Solving frustrated quantum many-particle models with convolutional neural networks. *Physical Review B: Condensed Matter and Materials Physics*.

[23] Hou F., Li B., Chong A. Y. L., Yannopoulou N., Liu M. (2017). Understanding and predicting what influence online product sales? a neural network approach. *Production Planning & Control*.

[24] Han S., Ren F., Wu C., Chen Y., Du Q., Ye X. (2018). Using the tensorflow deep neural network to classify mainland China visitor behaviours in Hong Kong from check-in data. *ISPRS International Journal of Geo-Information*.

[25] Zhang Y.-D., Dong Z., Chen X. (2019). Image based fruit category classification by 13-layer deep convolutional neural network and data augmentation. *Multimedia Tools and Applications*.

[26] Połap D., Włodarczyk-Sielicka M., Wawrzyniak N. (2021). Automatic ship classification for a riverside monitoring system using a cascade of artificial intelligence techniques including penalties and rewards. *ISA Transactions*.

